The article "MiR-506 Suppresses Tumor Proliferation and Invasion by Targeting FOXQ1 in Nasopharyngeal Carcinoma" was retracted in 2022. Reasons: duplicated images; signs of a paper mill; concerns about the data; concerns about the results or conclusions.

# MiR-506 Suppresses Tumor Proliferation and Invasion by Targeting FOXQ1 in Nasopharyngeal Carcinoma

**DOI:** 10.1371/journal.pone.0122851

**Published:** 2015-04-09

**Authors:** Zhanchi Zhang, Jun Ma, Guang Luan, Lin Kang, Yuhong Su, Yanan He, Feng Luan

**Affiliations:** 1 Department of Human Anatomy, Hebei Medical University, Shijiazhuang, PR China; 2 The Third Hospital of Hebei Medical University, Shijiazhuang, PR China; 3 Department of Otorhinolaryngology, The Third Hospital of Hebei Medical University, Shijiazhuang, PR China; Peking Union Medical College Hospital, CHINA

## Abstract

MiRNAs are small noncoding RNAs that play important roles in various biological processes including tumorigenesis. However, little is known about the expression and function of miR-506 in nasopharyngeal carcinoma (NPC). In this study, we showed that miR-506 was downregulated in nasopharyngeal carcinoma (NPC) cell lines and tissues. Ectopic expression of miR-506 dramatically suppressed cell proliferation, colony formation and invasion. Moreover, we identified the Forkhead box Q1 (FOXQ1) gene as a novel direct target of miR-506. MiR-506 exerts its tumor suppressor function through inhibition of the FOXQ1, which was involved in tumor metastasis and proliferation in various cancers. Furthermore, the expression of FOXQ1 is up-regulated in NPC cell lines and tissues. Taken together, our results indicate that miR-506 functions as a tumor suppressor miRNA in NPC and that its suppressive effects are mediated chiefly by repressing FOXQ1 expression.

## Introduction

Nasopharyngeal carcinoma (NPC) is a non-lymphomatous squamous cell carcinoma arising from epithelial cells located in the nasopharynx, which is low globally but high in southern China and Southeast Asia[1–3]. The characteristics are highly malignant local invasion and early distant metastasis, and 30–40% of NPC patients will develop distant metastases with poor prognosis[4–6]. NPC responds well to radiation therapy and adjuvant chemotherapy, however, the 5-year overall survival rate is still approximately 70%[7–9]. Therefore, an improved understanding of the mechanisms of NPC tumorigenesis is urgently needed for the development of more effective therapies for NPC.

MicroRNAs (miRNAs) are small non-coding RNAs (21–25 nucleotides) that regulate gene expression by causing mRNA cleavage or inhibition of mRNA translation by interaction with the 3’-untranslated region (3’-UTR) of the target gene mRNA[10–14]. Accumulated evidences prove that miRNAs play important regulatory roles in many critical biological processes including cell development, proliferation, differentiation, apoptosis, invasion, migration and so on[11, 15–19]. A large number of studies demonstrated that the gain or loss of miRNAs functions contribute to cancer development through the silencing of tumor suppressor genes and upregulation of oncogenes in various cancers such as breast cancer, gastric cancer, hepatocellular carcinoma and Ewing's sarcoma[20–25].

The article "MiR-506 Suppresses Tumor Proliferation and Invasion by Targeting FOXQ1 in Nasopharyngeal Carcinoma" was retracted in 2022. Reasons: duplicated images; signs of a paper mill; concerns about the data; concerns about the results or conclusions.

In our study, we identified that miR-506 was down-regulated in NPC cell lines and tissues, and miR-506 was further identified to be a tumor suppressor, as overexpression of miR-506 in NPC cell lines can inhibit cell proliferation and invasion by targeting Forkhead box Q1 (FOXQ1). Thus, our date suggest important roles of miR-506 in NPC pathogenesis and indicate its potential application in cancer therapy.

## Results

### The expression of miR-506 was lower in NPC cell lines and tissues

The expression of miR-506 was frequently decreased in NPC tissues compared with normal nasopharyngeal epithelial specimens (Fig 1A). Moreover, miR-506 was also down-regulated in all 4 NPC cell lines (5–8 F, 6-10B, CNE1 and CNE2) examined when compared with the nasopharyngeal epithelial cell line NP69 (Fig 1B).

**Fig 1:** The expression of miR-506 was lower in NPC cell lines and tissues. (A) qRT-PCR analysis was used to detect the expression of miR-506 in NPC tissues and normal nasopharyngeal epithelial specimens. (B) qRT-PCR analysis was used to detect the expression of miR-506 in all NPC cell lines (5–8 F, 6-10B, CNE1 and CNE2) and one nasopharyngeal epithelial cell line NP69. The expression of miR-506 was normalized to U6 snRNA. ***p<0.001.

### Overexpression of miR-506 inhibited NPC cell proliferation and colony formation

The highly up-regulated expression of miR-506 was confirmed by qPCR in both 5–8 F and 6-10B cell lines (Fig 2A). CCK-8 proliferation assay showed that overexpression of miR-506 repressed the 5–8 F and 6-10B cell lines proliferation when compared with those of scramble infected cells (Fig 2B and 2C). Colony formation assay also showed that overexpression of miR-506 inhibited the 5–8 F and 6-10B cell colony formation (Fig 2D).

**Fig 2:** Overexpression of miR-506 inhibited NPC cell proliferation and colony formation. (A) The highly up-regulated expression of miR-506 was confirmed by qPCR in both 5–8 F and 6-10B cell lines (B) Overexpression of miR-506 repressed the 5–8 F cell line proliferation when compared with those of scramble infected cells using CCK-8 proliferation assay. (C) Overexpression of miR-506 repressed the 6-10B cell line proliferation when compared with those of scramble infected cells using CCK-8 proliferation assay. (D) Colony formation assay also showed that overexpression of miR-506 inhibited both the 5–8 F and 6-10B cell colony formation. ** p<0.01, and ***p<0.001.

The article "MiR-506 Suppresses Tumor Proliferation and Invasion by Targeting FOXQ1 in Nasopharyngeal Carcinoma" was retracted in 2022. Reasons: duplicated images; signs of a paper mill; concerns about the data; concerns about the results or conclusions.

### Overexpression of miR-506 repressed invasion of NPC cells

To explore the function of miR-506 on motility of NPC cells, invasion assays were performed. As shown in Fig 3, we showed that the percentage of invasive cells was significantly lower in cells transfected with miR-506 mimic compared with those infected with scramble.

**Fig 3:** Overexpression of miR-506 repressed invasion of NPC cells. Invasion analysis has shown that the percentage of invasive cells was significantly lower in cells transfected with miR-506 mimic compared with those infected with scramble. ***p<0.001.

### MiR-506 directly targeted FOXQ1

As predicted by PicTar, there was complementarity between has-miR-506 and the FOXQ1 3’UTR (Fig 4A). The effect of miR-506 on the translation of FOXQ1 mRNA into protein was then assessed by using a luciferase reporter assay (Fig 4B). Over-expression of miR-506 remarkably repressed the luciferase activity of the reporter gene with the wild-type construct but not with the mutant FOXQ1 3’UTR construct in both 5–8 F and 6-10B cells, which indicates that miR-506 directly targeted the FOXQ1 3’UTR.Overexpression of miR-506 inhibited the protein and mRNA levels of FOXQ1 in both 5–8 F and 6-10B cells (Fig 4C and 4D).

**Fig 4:** MiR-506 directly targeted FOXQ1. (A) Predicted miR-506 target sequence in the 3’UTR of FOXQ1 (FOXQ1-3’-UTR-WT) and mutant containing 7 altered nucleotides in the 3’UTR of FOXQ1 (FOXQ1-3’-UTR-MUT). (B) The analysis of the relative luciferase activities of FOXQ1-WT, FOXQ1-MUT in the 5–8 F cells and 6-10B cells. (C) Western blot analysis of FOXQ1 expression in the 5–8 F and 6-10B cells transfected with miR-506 mimics or scramble. GAPDH was detected as a loading control. (D) qRT-PCR analysis of FOXQ1 mRNA expression in the 5–8 F and 6-10B cells after treatment with miRNA mimics or scramble. The expression of FOXQ1 was normalized to GAPDH. ***p<0.001.

### The tumor suppressor role of miR-506 was mediated by downregulating FOXQ1

We performed a gain-of-function assay to study the tumor suppressor role of miR-506 in NPC is mediated by repressing the expression of FOXQ1. FOXQ1 expression vectors, pcDNA-FOXQ1 was used to restore FOXQ1 expression (Fig 5A). As shown in Fig 5B, the inhibitory role of miR-506 in proliferation was rescued under the condition of overexpression of FOXQ1. Moreover, similar results could be observed when cell invasion assays were carried out (Fig 5C).

**Fig 5:** The tumor suppressor role of miR-506 was mediated by downregulating FOXQ1. (A) Western blot analysis showed that pcDNA-FOXQ1 can restore FOXQ1 expression. The expression of FOXQ1 was normalized to GAPDH. (B) The inhibitory role of miR-506 in proliferation was rescued under the condition of overexpression of FOXQ1. (C) The inhibitory role of miR-506 in invasion was rescued under the condition of overexpression of FOXQ1. *p<0.05, ** p<0.01, ***p<0.001

The article "MiR-506 Suppresses Tumor Proliferation and Invasion by Targeting FOXQ1 in Nasopharyngeal Carcinoma" was retracted in 2022. Reasons: duplicated images; signs of a paper mill; concerns about the data; concerns about the results or conclusions.

### The expression of FOXQ1 was higher in NPC cell lines and tissues

The expression of FOXQ1 was frequently increased in NPC tissues compared with normal nasopharyngeal epithelial specimens (Fig 6A). Moreover, FOXQ1 was also down-regulated in all 4 NPC cell lines (5–8 F, 6-10B, CNE1 and CNE2) examined when compared with the nasopharyngeal epithelial cell line NP69 (Fig 6B).

**Fig 6:** The expression of FOXQ1 was higher in NPC cell lines and tissues. (A) qRT-PCR analysis was used to detect the expression of FOXQ1 in all NPC cell lines (5–8 F, 6-10B, CNE1 and CNE2) and one nasopharyngeal epithelial cell line NP69. (B) qRT-PCR analysis was used to detect the expression of FOXQ1 in NPC tissues and normal nasopharyngeal epithelial specimens. The expression of FOXQ1 was normalized to GAPDH.

## Discussion

In this study, we reported for the first time that miR-506 was markedly down-regulated in NPC clinical specimens and cell lines. The over-expression of miR-506 repressed the proliferative and invasive capacities of NPC cells. Moreover, we identified that the expression of FOXQ1 mRNA and protein was down-regulated after transfected miR-506 mimic in NPC cells by qPCR and western blot. FOXQ1 was identified as a new direct and functional target of miR-506 by using dual luciferase assay. The ectopic expression of FOXQ1 could rescue partially the suppressive effect of miR-506, and we also found FOXQ1 expression is up-regulated in NPC tissues. Our study suggested that miR-506 acts as a novel proliferation and metastasis suppressor by targeting FOXQ1 in NPC.

Recently, miRNAs have been shown to be crucial in maintenance of normal cellular function, and the dysregulation of miRNAs expression can result in tumor progression and cancer initiation[26–28]. Accumulating evidence indicated that miR-506 is abnormally expressed and has been implicated in various tumors[29–33]. Liu et al[29]. has reported that miR-506 functions as a tumour suppressor in ovarian cancer. miR-506 regulates cell proliferation and senescence by directly targeting its binding sites on the 3’-UTRs of CDK4 and CDK6. Moreover, miR-506 upregulation occurs in 83% of lung cancer patients (156 cases), and its expression highly correlates with ROS[34]. Ectopic expression of miR-506 inhibits NF-kB p65 expression, induces ROS accumulation and then activates p53 to suppress lung cancer cell viability. However, miR-506 has been demonstrated to act as an oncogene in melanomas and can confer chemoresistance in colon cancer[35]. The expression pattern of miR-506 is different, even contradictory, in different types of malignant carcinoma, suggesting the complex role of miR-506 in cancer progression. In our study, we identified that the expression of miR-506 was significantly down-regulated in NPC tissues and cell lines. Overexpression of miR-506 significantly repressed cell proliferation and invasion in both 5–8 F and 6-10B cell lines. These data suggest a tumor-inhibiting role of miR-506 in NPC cells.

The article "MiR-506 Suppresses Tumor Proliferation and Invasion by Targeting FOXQ1 in Nasopharyngeal Carcinoma" was retracted in 2022. Reasons: duplicated images; signs of a paper mill; concerns about the data; concerns about the results or conclusions.

Our mechanistic investigations revealed that miR-506 exerts its influence on the proliferation and invasion of NPC by directly targeting its binding sites on the 3’-UTRs of FOXQ1. Bioinformatics tools predicted FOXQ1 to be a theoretical target gene of miR-506. In this report, we verified FOXQ1 as a direct target of miR-506 using luciferase reporter gene assay. Moreover, overexpression of miR-506 could repress both the mRNA and protein levels of FOXQ1. Restoring the expression of FOXQ1 can reverse the suppressive effects of miR-506. In addition, we found that the expression of FOXQ1 was up-regulated in NPC tissues and cell lines. These data suggest that FOXQ1 is a direct and functional target of miR-506 in NPC cells.

FOXQ1, also known as HFH1, is a member of the FOX gene family and contains the core DNA binding domain; whereas the flanking wings of FOXQ1 contribute to its sequence specificity[36–38]. FOX genes are involved in many critical biological processes such as cell cycle regulation, embryonic development, cell signaling, tissue-specific gene expression and tumorigenesis[39–42]. Recent studies have reported that FOXQ1 was involved in tumor metastasis and proliferation in glioblastoma, colorectal cancer, hepatocellular carcinoma and breast cancer[42–44]. Previous results implied that FOXQ1 was a prognostic marker for gastric cancer and hepatocellular carcinoma patients[42]. Recently, Peng et al[45]. showed that FOXQ1 was overexpressed in NPC cell lines and tissues and FOXQ1 expression increased with clinical stage, T stage. However, the underlying mechanisms are unclear. Our data showed that the ability of miR-506 to target FOXQ1 may provide one such mechanism of post-transcriptional control of FOXQ1.

In conclusion, our results suggest that the expression of miR-506 is down-regulated in NPC tissues and cell lines, and functions as a novel tumor suppressor to repress the proliferation and invasion of NPC cells by targeting FOXQ1. Therefore, miR-506 may be a novel molecular therapeutic target for the treatment of NPC.

## Materials and Methods

### Ethics statement

All of these patients agreed to participate in the study and gave written informed consent. Both this study and consent were approved by the ethical board of The Third Hospital of Hebei Medical University and complied with the Declaration of Helsinki.

The article "MiR-506 Suppresses Tumor Proliferation and Invasion by Targeting FOXQ1 in Nasopharyngeal Carcinoma" was retracted in 2022. Reasons: duplicated images; signs of a paper mill; concerns about the data; concerns about the results or conclusions.

### Cell line and tissue specimens

Human nasopharyngeal carcinoma cell lines such as 5–8 F (an NPC cell line with high tumorigenic and metastatic ability), 6-10B, CNE1 and CNE2 (Cell Bank of Chinese Academy of Science, Shanghai, China) were cultured in RPMI-1640 medium (HyClone, Thermo scientific Inc, China) according to previous studies’ method[45, 46]. The above cell lines were supplemented with 10% fetal bovine serum (FBS, HyClone, Thermo scientific Inc, China). Primary NPC biopsy specimens and normal biopsies of the nasopharynx were collected from our Hospital. No patients had received blood transfusion, radiotherapy, or chemotherapy before surgery.

### Quantitative real-time PCR (qPCR) assay

Total RNA was purified with Trizol Reagent (Invitrogen) from cells or tissues. The expression levels of miRNAs were determined by SYBR Green quantitative PCR amplifications performed on the 7500 Fast System real-time PCR cycler (Applied Biosystems, USA). The primers used for PCR amplification were shown as S1 Table. All mRNA quantification data were normalized to GAPDH and miRNA quantification data were normalized to U6.

### Oligonucleotides and Transfection

MiR-506 mimics and scramble were chemically synthesized from Dharmacon. Cells were transfected using Lipofectamine 2000 reagent (Invitrogen) following to the manufacturer’s instructions. Transfection complexes were prepared according to the manufacturer's instructions and added directly to the cells.

### Western blot analysis

Western blotting was carried out as described previously[47, 48]. Total cell or tissue proteins were separated using 10% SDS-PAGE gels, and transferred to PVDF (polyvinylidene fluoride) membranes (Millipore). Then, the membranes were incubated with mouse monoclonal Anti- FOXQ1 antibody (Sigma-Aldrich) or Anti-GAPDH antibody (Cell Signaling Technology). Anti-GAPDH antibody was from Santa Cruz Biotechnology. Bands were detected with chemiluminescence.

### Cell proliferation and colony formation assays

Cell proliferation was measured using a Cell Counting Kit-8 (CCK-8, Dojindo Molecular Technologies, Kumamoto, Japan) following the manufacturer’s instructions. After transfection, the cells were cultured for 24, 48 and 72 hours. For colony formation assay, cells were seeded into each well of 6-well plates. The cells were fixed using 70% ethanol and stained with 1% crystal violet solution for 20 min to visualize colonies for counting after 10 days in culture.

### Luciferase reporter assay

Cells at 70% confluence in a 96-well plate were transfected with 0.01 μg Renilla and 0.1 μg firefly using 0.25 μl of transfection reagent. Cell extracts were prepared 48 h after co-transfection, and the luciferase activity was detected using a Luciferase Reporter Assay System kit (Promega, Madison, WI, USA). The mean values were detected, and the firefly luciferase activity was normalized to the Renilla luciferase activity.

The article "MiR-506 Suppresses Tumor Proliferation and Invasion by Targeting FOXQ1 in Nasopharyngeal Carcinoma" was retracted in 2022. Reasons: duplicated images; signs of a paper mill; concerns about the data; concerns about the results or conclusions.

### Cell invasion assay

At 48 hours after transfection, cells were seeded onto the basement Matrigel-coated membrane matrix (BD Biosciences) present in the insert of a 24-well culture plate. Fetal bovine serum was added to the lower chamber as a chemoattractant. After a further 48 hours, the noninvading cells were gently removed with a cotton swab. Invasive cells located on the lower side of the chamber were stained with Crystal Violet and counted.

### Statistical analysis

Data were expressed as means ±SD (standard deviation). Two treatment groups were compared by the unpaired Student’s t test; one-way ANOVA was performed for serial analysis. A value of P<0.05 was considered statistically significant.

## Supporting Information

S1 Table Primer sequence. (DOCX)
